The article "Knowledge, Attitude, and Practice regarding Testicular Cancer and Testicular Self-Examination among Male Students Pursuing Bachelor's Degree in Bharatpur Metropolitan City, Chitwan, Nepal" was published in 2021. Journal: Biomed Res Int.

# Knowledge, Attitude, and Practice regarding Testicular Cancer and Testicular Self-Examination among Male Students Pursuing Bachelor's Degree in Bharatpur Metropolitan City, Chitwan, Nepal

**DOI:** 10.1155/2021/1802031

**Published:** 2021-08-31

**Authors:** Radha Dhakal, Samkisha Paudel, Dipesh Paudel

**Affiliations:** ^1^Shree Medical and Technical College, Bharatpur, Nepal; ^2^Chitwan Medical College, Bharatpur, Nepal

## Abstract

**Background:**

Testicular cancer is a malignant tumor of the testicles, the male reproductive organs that produce sperm and testosterone. It is one of the most common cancers in young men. This form of cancer can be easily diagnosed by self-examination of testicles and is curable if detected early. Periodic self-examination must be performed for early detection. Due to lack of knowledge on testicular cancer and testicular self-examination techniques, patients can potentially miss early detection. This study is aimed at assessing the knowledge, attitude, and practice regarding testicular cancer and testicular self-examination among male college students pursuing a Bachelor's degree.

**Methods:**

A web-based cross-sectional analytical study was adopted to assess the knowledge, attitude, and practice of testicular cancer and testicular self-examination among male college students pursuing a Bachelor's degree and living in Bharatpur Metropolitan City in the Chitwan District of Nepal. The snowball sampling technique was employed to identify the eligible participants. Collected data were entered in SPSS version 22 and analyzed by using the Chi-square test, Pearson's correlation, and binary logistic regression.

**Results:**

Out of 402 respondents, majority (56.7%) had poor knowledge regarding testicular cancer and testicular self-examination and only 11.4% had performed testicular self-examination. The majority (67.2%) of the respondents had shown an unfavorable attitude towards testicular cancer (TC) and testicular self-examination (TSE). There was a significant association between the level of knowledge and marital status 4.516 (1.962-10.397) and ethnicity 2.606 (1.443-4.709). Likewise, age 0.396 (0.191-0.821) and marital status 0.347 (0.156-0.775) have been significantly associated with testicular self-examination practice. Regarding favorable attitude, age 0.362 (0.186-0.706) and sources of information from mass media 2.346 (1.328-4.143) have been associated significantly.

**Conclusion:**

The study finding shows that the knowledge on testicular cancer and testicular self-examination was low. Due to lack of knowledge and trainings, the potential opportunities for early detection of testicular cancer are missed substantially. Periodic testicular self-examination is vital for early detection of testicular cancer. Hence, it is crucial to implement massive educational campaigns and trainings on testicular cancer and testicular self-examination techniques among young male groups.

## 1. Background

Testicles are the vital organs of the male reproductive system. They produce sperm and testosterone which play a key role in male sexual development. The most common type of testicular cancer is germ cell testicular cancer that starts in the testicles [1]. Testicular cancer is rare, but it is one of the most commonly diagnosed cancers in young adult men, particularly between the 20- and 40-year age group [2]. The risk factors for testicular cancer include undescended testicle, family history of testicular cancer, HIV infection, carcinoma in situ of the testicle, having had testicular cancer before, and body size. The common sign of cancer is painless masses on testicles [3].

More socioeconomically developed countries had a higher incidence of testicular cancer with lower mortality—Western (8.7%) and Northern European (7.2%) countries had the highest incidence rate. The incidence rates were markedly increased in Southern European countries with an average annual percent change of 6.8% in Croatia and 6.1% in Spain [4]. The number of cases of testicular cancer diagnosed each year in the United Kingdom (UK) has roughly doubled since the mid-1970s, with around 2300 new cases each year [1]. The incidence of testicular cancer has been increasing in the United States (US) with an estimated number of new cases of 9,470, and about 440 deaths in 2021 [2]. In Nepal, very few testicular cancer studies have been conducted. Out of 70 abnormal testicular mass cases, 11.4% (8/70) were diagnosed as malignant testicular tumors [5].

Testicular self-examination (TSE) is a screening technique that involves inspection of the appearance and palpation of the testes to detect any changes from normal [6]. Self-examination of the testes is important for the early detection of testicular cancer. The most common method of early detection is performing a monthly exam. Upon reaching puberty, all men should conduct a monthly testicular self-exam [7]. Testicular cancer is a form of cancer, which is easily diagnosable by TSE and is 96% curable if detected early [8]. Testicular self-examination is an easy way for male adults to check their testicles to make sure there are no unusual lumps or bumps which can be the first sign of testicular cancer [9].

There has been much attention given to awareness of breast cancer and breast self-examination. Only few studies have been conducted on knowledge, attitude, and practice (KAP) towards testicular cancer (TC) and testicular self-examination (TSE). It is important to examine the KAP towards TC and TSE among the male adults that belong to the risky age group (20-40 years) to understand the level of awareness. Hence, this study was planned to assess KAP on TC and TSE among college students pursuing a Bachelor's degree.

## 2. Method

### 2.1. Study Design, Setting, and Population

A web-based cross-sectional analytical study design was undertaken to assess the knowledge, attitude, and practice of testicular cancer and testicular self-examination among male college students pursuing a Bachelor's degree. The research was carried out in Bharatpur Metropolitan City in the Chitwan District, which is located in the central-southern part of Nepal. There are 39 higher secondary schools and more than 10 nonmedical degree colleges in Bharatpur [10].

### 2.2. Sample Size

The sample size was calculated based on 61% prevalence [11]:

(1) $$\begin{array}{c} \text{Sample size }\left(n\right)=Z\alpha^{2}*p*\frac{q}{e^{2}}, \end{array}$$

where *Zα* = 1.96, error (*e*) = 5% = 0.05%, prevalence taken for calculation is 61%, *q* = (1 − *p*) = 1 − 0.61 = 0.39.

By using formula (1), the sample size is calculated as follows:

(2) $$\begin{array}{c} \text{Sample size }\left(n\right)=\frac{{\left(1.96\right)}^{2}*0.61*0.039}{{\left(0.05\right)}^{2}}=\frac{0.91391}{0.0025}=365.56\;\left(10\%\text{nonresponse error}\right)=365+37=402. \end{array}$$

Hence, a sample size of 402 was considered for the study.

### 2.3. Sampling Technique

The nonprobability snowball or networking sampling technique was employed to identify the eligible participants. This technique was chosen to suit the data collection during a pandemic when colleges were closed for an uncertain period. At first, the researchers prepared a list of Bachelor degree colleges in Bharatpur Metropolitan City and their contact numbers. This started with the researchers first approaching the students in their network. Currently, most of the colleges have taken classes via online platforms and have created their private groups in Viber, WhatsApp, Messenger, and Emails for communication. In the different online platforms of Bachelor's degree students, participants were invited to participate in this survey and further requested to pass the survey to other eligible participant(s) in their network.

### 2.4. Validity and Reliability

The questionnaire was developed by the researchers based on an extensive literature review and consultation with the subject matter experts. To increase the content validity, the questionnaire was first prepared in English and then translated into Nepali language and backtranslated to English. Pretesting of the questionnaire was done in 10% of the population (*n* = 40) in a similar setting. Internal consistency of the questionnaire was ensured based on Cronbach's alpha value, where Cronbach's alpha coefficient of knowledge questionnaire was 0.837, indicating acceptable internal consistency. Depending on the pretest, essential modifications and adjustments of the questionnaire were addressed through expert consultation.

### 2.5. Data Collection Procedure

The online administered questionnaire was preferred to reach out to the participants quickly and effectively during the pandemic. The principal investigator created the questionnaire as a Google Form and shared it online to the willing participants by networking with them in different online sharing platforms like Messenger, Viber, WhatsApp, and Emails of male college students pursuing a Bachelor's degree in various colleges of Bharatpur Metropolitan City.

### 2.6. Data Analysis Procedure

Fully completed questionnaires were extracted from Google Forms and exported to Microsoft Excel 2016 for cleaning and coding. All data received from the online system was checked for completeness and then imported, entered, analyzed, and interpreted by using IBM SPSS version 22 software. Descriptive statistics methods (in terms of frequency and percent) and inferential statistics (Pearson's chi-square test, logistic regression, and correlation) were used to determine the association.

### 2.7. Ethical Considerations

Ethical norm was considered and followed throughout the study. The ethical approval was taken from Shree Medical and Technical College and SMTC-IRC-20210109-12. Informed written consent was taken from the participant before data collection. No personal information like name, email id, address, or license number was collected. All submitted forms were collected in the email of the principal investigators only. The participation of the respondents in the study was voluntary, and they were well informed that they could withdraw from the study at any time if they wish. Confidentiality and anonymity were maintained by coding the serial numbers instead of the name of the subject.

### 2.8. Operational Definition

#### 2.8.1. Knowledge of Testicular Cancer

It refers to the facts or information like meaning, risk factors, signs and symptoms, treatment, and prevention that respondents have regarding testicular cancer. It was categorized as good knowledge and poor knowledge based on the mean score.

#### 2.8.2. The Attitude of Testicular Cancer

It refers to the opinion, feeling, thought, and the idea that the respondent has towards testicular cancer. It was assessed by the score obtained through the attitude (Likert) scale. The scale included 8 attitude items with a total score of 40; a score of >24 was considered to reflect a favorable attitude, and a score ≤ 24 as unfavorable attitude. The scoring procedure for attitude was based on a 5-point Likert scale where positive statements were scored as strongly agree=5, agree=4, neutral=3, disagree=2, and strongly disagree=1. Reverse scoring was done for negative statements.

#### 2.8.3. The Practice of Testicular Self-Examination

It refers to the act of doing or performing testicular self-examination by respondents. It was measured by asking yes or no questions.

#### 2.8.4. Male Bachelor Degree Students

This group refers to those individuals who are studying in Bachelor degree colleges (nonmedical) of Bharatpur Metropolitan City, Chitwan.

## 3. Results

### 3.1. Sociodemographic Characteristics of the Respondents

Table 1 shows that out of 402 respondents, the majority (61.4%) of the respondents were in the age group of 21-25 years and 1.2% were in the age group of above 35 years. The mean age of the respondents was 23.51 years. The minimum age was 16 years, and the maximum age was 37 years. Concerning marital status, the majority (84.3%) were unmarried, whereas a few of them (15.7%) were married. Regarding ethnicity, majority (71.9%) were Brahmin/Chettri. Consequently, about religion, most of the respondents (89.6%) followed Hinduism and a few (0.7%) followed Islam. At the same time, concerning education, most of the respondents (58%) were at 4th year of their Bachelor's degree, whereas just 11.4% of the respondents were at the 2nd year, respectively. Most importantly, the family history of testicular cancer was not found in majority of the respondents (98.0%). Likewise, 87.3% of the respondents did not have any sort of testicular abnormality. Furthermore, the source of information on testicular cancer for a considerable number of respondents, i.e., 68.9%, turned out to be mass/media.

### 3.2. Respondents' Knowledge regarding Testicular Cancer and Testicular Self-Examination

Table 2 shows that 39.3% of the respondents knew the meaning of testicular cancer. Regarding the age group at high risk of developing testicular cancer, 38.3% gave the correct response. Majority of the respondents (45.8%) gave a correct response on the most common signs and symptoms of testicular cancer being a painless lump in the testicles. Concerning risk factors, 95.8% gave a correct response on multiple sex partner which is not a risk factor of TC, and 54.7% gave a correct response on positive family history which is a risk factor of TC. Regarding the best way to treat testicular cancer, 80.3% gave the correct response on early detection. Furthermore, when asked about the frequency of testicular self-examination, only 14.7% of the respondents gave the correct response—once a month. At a glance, we can also see in Table 2 that 16.7% of the respondents gave the correct response for the most common complications of testicular cancer. Nevertheless, we can also interpret that the majority (95.3%) of the respondents know the fact that regular testicular self-examination could be the best way to prevent testicular cancer.

### 3.3. Distribution of Respondents according to Practice of Testicular Self-Examination

Table 3 shows that out of 402 respondents, 88.6% responded that they do not practice TSE and 11.4% responded to have practiced testicular self-examination. When asked about how often they need to perform TSE to those who said they practice TSE, the majority (37.0%) said that they do it once a month and at least 17.4% said once in six months. Consequently, when asked about the reasons for not doing TSE to those who said they do not practice TSE, majority (58.4%) of the respondents said that they do not know how to perform TSE, while only 5.9% said that they think that doing TSE is a sin or taboo.

### 3.4. Respondents' Attitude regarding Testicular Cancer and Testicular Self- Examination

Table 4 shows that 40.7% of the respondents strongly agree with the fact that TSE helps in the early detection of testicular cancer, while 33.8% of the respondents disagree that testicular cancer has no cure. At the same time, surprisingly, 35.8% of the respondents strongly agree that TSE is a form of masturbation. In addition, 39.1% of the respondents remained neutral with the fact that men having testicular cancer are completely infertile. However, as per Table 4, it is clear that 33.6% of the respondents gave a neutral response to the statement that TSE often strikes men at their age. On the contrary, 32.8% of the respondents gave the neutral view that TSE should be done once a month regularly. Likewise, 43.5% of the respondents had a neutral response that TSE should be done during the shower or shortly after the shower. And last but not the least, 24.4% of the respondents agreed that testicular cancer is a common cancer.

### 3.5. Respondents' Level of Knowledge, Attitude, and Practice regarding Testicular Cancer and Testicular Self-Examination

Table 5 shows that the majority (56.7%) of the respondents had poor knowledge regarding testicular cancer, and likewise, 43.3% had good knowledge regarding testicular cancer. Regarding the attitude, majority (67.2%) of the respondents had an unfavorable attitude regarding testicular cancer and testicular self-examination, while on the contrary, 32.8% had an unfavorable attitude regarding testicular cancer and testicular self-examination. Further, practice was leveled as “performed” and “not performed” testicular self-examination where majority (88.6%) of the respondents have not performed and (11.4%) have performed testicular self-examination.

### 3.6. Association between KAP Levels regarding Testicular Cancer and Testicular Self-Examination and Sociodemographic Variables

Table 6 shows the association between the level of KAP with testicular cancer and testicular self-examination and sociodemographic variables. Knowledge was significantly associated with age (*p* = 0.008), marital status (*p* = 0.016), ethnicity (*p* = 0.024), education (*p* < 0.001), history of testicular abnormalities (*p* < 0.001), and source of information from parents and teachers (*p* < 0.001). Likewise, attitude was significantly associated with age (*p* < 0.001), ethnicity (*p* = 0.002), family history (*p* = 0.046), history of testicular abnormalities (*p* = 0.031), and sources of information from mass media, parents, and teachers (*p* < 0.001). Practice was significantly associated with age (*p* = 0.001), marital status (*p* < 0.001), history of testicular abnormalities (*p* = 0.015), source of information from health workers (*p* < 0.001), sex education (*p* < 0.001), and mass media (*p* = 0.0073).

### 3.7. Logistic Regression Analysis for Sociodemographic Factors Associated with KAP regarding Testicular Cancer and Testicular Self-Examination

Table 7 shows that marital status 4.516 (1.962-10.397), ethnicity 2.606 (1.443-4.709), education 2.568 (1.549-4.258), and history of testicular abnormality 12.827 (4.850-33.924) have been associated with good knowledge. Regarding favorable attitude, age 0.362 (0.186-0.706), ethnicity 0.399 (0.218-0.728), history of testicular abnormality 0.426 (0.189-0.960), source of information from mass media 2.346 (1.328-4.143), and parents and teachers 1.956 (1.162-3.291) have associated significantly. Age 0.396 (0.191-0.821) and marital status 0.347 (0.156-0.775) have been associated with testicular examination practice.

### 3.8. Correlation between KAP Scores

Table 8 shows that the Pearson correlation test revealed a statistically significant negative correlation between knowledge and practice (*r* = −0.301; *p* < 0.001) and a positive correlation between practice and attitude (*r* = 0.100; *p* = 0.045) and no significant correlation between knowledge and practice (*r* = −093; *p* = 0.061).

## 4. Discussion

Several studies have been conducted on knowledge, attitudes, and practice towards TC and TSE among university students. In this study, most of the respondents have poor knowledge, attitude, and practice towards TC and TSE. There were significant associations between KAP levels and some sociodemographic factors like age (*p* = 0.008), marital status (*p* = 0.016), education (*p* < 0.001), history of testicular abnormalities (*p* < 0.001), and source of information from parents and teachers (*p* < 0.001). These findings are supported by the study conducted in Northeast Ethiopia [8], Turkey [12], and Nigeria [13] as well.

### 4.1. Knowledge towards TC and TSE

In the current study, out of 402 respondents, the majority (56.7%) of the respondents had poor knowledge. This finding is in line with other study findings from (53%) Ethiopia [14] and (53%) Bahrain [15]. This was lower than other related studies conducted (90%) in London [16] and (61.36%) in Saudi Arabia[11], although it is greater than the study findings (44%) from Turkey [17] and (41.2%) Uganda [6]. This variation might be due to their difference in sociodemographic characteristics, knowledge questions, study setting, and study design. In this study, 39.3% of the respondents knew the meaning of testicular cancer. This finding is supported by the study conducted (44%) in Northeast Ethiopia [8]. In the current study, regarding the high-risk age group for developing testicular cancer, only 38.3% gave the correct response, i.e., the 15–40-year age group. This is supported by the study conducted (32.7%) in Nigeria [13]. It is a higher figure (28.8%) than the study conducted (28.8%) in Northeast Ethiopia [8] and lower than (68.5%) in the USA [18]. This variation might be due to the higher awareness and screening practice in developed countries compared to that of underdeveloped or developing countries. Likewise, in this study, 45.8% knew the most common signs and symptoms of TC, which is a higher figure than the study findings (23.56%) of Saudi Arabia [11], same line with the study findings (38.3%) of Turkey [17], and lower than the study findings (15%) from Bahrain [14]. In this study, regarding risk factors, 54.7% gave correct responses on family history, 58% on age, and 62.8% on prior trauma, and these findings are in contrast with the findings of Saudi Arabia which [11] shows family history of TC 29.38%, age 14.06%, and prior trauma 38.19%. In this study, 14.7% of the respondents gave the correct response on the frequency of testicular self-examination, which is comparable to the study conducted in (15.3%) Nigeria [19]. In this study, 16.1% of the respondents gave the correct answers regarding the most common complications, while 95.3% had good knowledge regarding prevention.

### 4.2. Practice regarding TSE

In this study, only 11.4% of the respondents practiced testicular self-examination, and this finding is similar to the study done in (11.38%) Saudi Arabia [11]. This was lower than other related studies conducted (66.7%) in Malaysia [20], (23.6%) Uganda [17], (21.5%) Northeast Ethiopia [11], and (22%) London [16], although it is greater than the study conducted (5.8%) in Bahrain [15]. These variabilities might be due to the study population, the number of practice questions, and the level of awareness of respondents on TC and TSE. In this study, 37.0% said that they do it once a month. This finding is supported by the study done in (36.45%) the USA [6], and it is higher than other related studies done (26.5%) in Ethiopia [8], (15.3%) Nigeria [12], and (6%) Bahrain [15]. Consequently, 58.4% of respondents said that they do not know how to perform TSE, which is lower than the study done in (73%) Bahrain [15], (83.4%) Turkey [18], and (62%) Ethiopia [14] and higher than the study findings (31.5%) from Uganda [6]. In this study, only 5.9% said that they think that doing TSE is a sin or taboo. These findings are supported by the studies done in (3.3%) Ethiopia [13] and (6.1%) Turkey [18].

### 4.3. Attitude towards TC and TSE

In this study, most of the respondents (67.2%) had unfavorable attitudes. This finding is higher than other related studies done (51.2%) in Northwest Ethiopia [8] and (30.8%) Nigeria [19]. This might be due to the variation in attitude scale, scoring technique, and level of knowledge. In this study, 47.0% of respondents strongly agreed that TSE helps in early detection, which is a very comparable figure with the study done (42.7%) in Turkey [21]. In this study, 33.8% of the respondents disagree that testicular cancer has no cure, and this finding is supported by the study done (47.31) in Saudi Arabia [11]. Similarly, in this study, 35.8% of the respondents said that TSE is a form of masturbation which is a higher figure than that in the study done (14%) in south Nigeria [22]. In addition, 39.1% of the respondents remained neutral to the fact that men having testicular cancer are completely infertile; however, 58.9% of the respondents agreed with the study done in London [16]. Likewise, in this study, 33.6% gave a neutral response with the statement that TC often strikes men at any age; however, 61.3% disagreed with the study done in Turkey [21]. In this study, 32.8% of the respondents gave neutral responses on the TSE done once in a month, which is a slightly lower figure than the study conducted (55.7%) in Turkey [21]. In this study, 43.5% of the respondents gave a neutral response on whether TSE should be done during the shower or shortly after a shower which is (65.7%) a lower figure than the study conducted in Turkey [21]. 32.8% gave a neutral response on the statement that TC is a common cancer and many men go through it, which disagrees with the study findings where 55.7% agreed in Turkey [21]. This study design included only 402 students. More representative students could not be reached because of the study design and sampling technique. The study was conducted online, and those who did not have access to the internet could not get a chance to enroll in the study. Therefore, the findings of this study cannot be generalized to other populations. Despite this limitation, this study contributes to the literature on the knowledge, attitudes, and practice of male college students pursuing a Bachelor's degree regarding testicular cancer and testicular self-examination.

## 5. Conclusion

This study revealed that the overall knowledge, practices, and attitude towards testicular cancer and testicular self-examination among male college students pursuing a Bachelor's degree were very low. This might be due to the sampling methods where the sample may not represent the population. However, knowledge and attitude are not the only factors for better practice. Due to lack of knowledge on testicular cancer and testicular self-examination techniques, potential opportunity for early detection of testicular cancer is missed. It is necessary to implement education campaigns, awareness programs, and testicular self-examination trainings among high-risk male groups.

## Figures and Tables

**Table 1:** Sociodemographic characteristics of the respondent (*n* = 402).

Characteristics	Category	Frequency (%)
Age in group	16-20	60 (14.9)
	21-25	247 (61.4)
	26-30	81 (20.2)
	31-35	9 (2.2)
Mean = 23.6294; Sd = 3.20916; min = 16.00; max = 37.00	Above 35	5 (1.3)
Marital status	Unmarried	339 (84.3)
	Married	63 (15.7)
Ethnicity	Dalit	6 (1.5)
	Janajati	67 (16.7)
	Madhesi	15 (3.7)
	Muslim	3 (0.7)
	Brahmin/Chettri	289 (71.9)
	Others (Giri, Puri, Thakuri)	22 (5.5)
Religion	Hinduism	360 (89.6)
	Buddhism	28 (7.0)
	Christianity	11 (2.7)
	Islam	3 (0.7)
Education level	Bachelor 1st year	58 (14.4)
	Bachelor 2nd year	46 (11.4)
	Bachelor 3rd year	65 (16.2)
	Bachelor 4th year	233 (58)
Family history of testicular cancer	Yes	394 (98%)
	No	8 (2%)
History of testicular abnormality	Yes	51 (12.7)
	No	351 (87.3)
Sources of information	Health worker	146 (20.9)
	Sex education	139 (19.9)
	Mass media	277 (68.9)
	Parents/teacher	136 (19.5)

**Table 2:** Respondents' knowledge regarding testicular cancer and testicular self-examination (*n* = 402).

Knowledge items	Correct response	Frequency (%)
Meaning of testicular cancer	Painless lump in testicles	158 (39.3)
Age group at risk for testicular cancer	16-40	154 (38.3)
Most common signs and symptoms	Painless lump in testicles	184 (45.8)
Risk factors of testicular cancer	Family history (yes)	220 (54.7)
	Multiple sex partner (no)	271 (67.4)
	Age (yes)	233 (58)
	Multiple children (no)	385 (95.8)
	Prior trauma to the testis (yes)	253 (62.9)
Best way to treat testicular cancer	Early detection	323 (80.3)
Frequency of doing a testicular self-examination	Once in a month	59 (14.7)
The most common complication of testicular cancer	Develop other cancer	67 (16.7)
Best way to prevent testicular cancer	Regular TSE	383 (95.3)

**Table 3:** Distribution of respondents according to practice of testicular self-examination (*n* = 402).

Practice item	Response	Frequency (%)
Testicular self-examination	Performed	46 (11.4)
	Not performed	356 (88.6)
If performed frequency (*n* = 46)	Once in a monthly	17 (37.0)
	Once in three months	12 (26.1)
	Once in six months	8 (17.4)
	Feel discomfort	9 (19.6)
Reason for not performing (*n* = 356)	Fear of result	25 (7.0)
	Not complaining	105 (29.5)
	Not knowing	208 (58.4)
	Not caring	45 (12.6)
	Feeling sinful	21 (5.9)

**Table 4:** Respondents' attitude regarding testicular cancer and testicular self-examination (*n* = 402).

SN	Statements	SA	A	N	D	SD
1.	TSE helps in the early detection of testicular cancer.	163 (40.6)	107 (26.6)	52 (12.9)	36 (9.0)	44 (10.9)
2.	Testicular cancer has no cure.	24 (6)	23 (5.7)	116 (28.9)	136 (33.8)	103 (25.6)
3.	TSE is a form of masturbation.	144 (35.8)	82 (20.4)	106 (26.4)	46 (11.4)	24 (6.0)
4.	Men having testicular cancer are completely infertile.	46 (11.4)	91 (22.6)	157 (39.1)	82 (20.4)	26 (6.5)
5.	Testicular cancer often strikes men my age.	36 (8.9)	82 (20.4)	135 (33.6)	114 (28.4)	35 (8.7)
6.	TSE should be done once a month regularly.	73 (18.2)	121 (30.1)	132 (32.8)	52 (12.9)	24 (6)
7.	TSE should be done in the shower or shortly after the shower.	32 (8)	39 (9.6)	175 (43.5)	106 (26.4)	50 (12.5)
8.	Testicular cancer is a common cancer. Many men go through it.	63 (15.6)	98 (24.4)	132 (32.8)	71 (17.7)	38 (9.5)

**Table 5:** Respondents' level of knowledge, attitude, and practice regarding testicular cancer and testicular self-examination (*n* = 402).

Variables	Frequency (%)	Mean score (SD)	Minimum score	Maximum score
Level of knowledge		6.4005 (1.565)	2.00	10.00
Good	174 (43.3)			
Poor	228 (56.7)			
Level of attitude		24.943 (4.470)	8.00	40.00
Favorable	132 (32.8)			
Unfavorable	270 (67.2)			
Level of practice				
Performed	46 (11.4)			
Not performed	356 (88.6)			

**Table 6:** Association between KAP levels regarding testicular cancer and testicular self-examination and sociodemographic variables.

		Level of knowledge			Level of attitude			Level of practice	*n* = 402	
Variables	Category	Good (%)	Poor (%)	*p* value	Favorable (%)	Unfavorable (%)	*p* value	Performed (%)	Not performed (%)	*p* value
Age in group	25 years	125 (39.8)	189 (60.2)		118 (37.6)	196 (62.4)		27 (8.6)	287 (91.4)	
	25 years	49 (55.7)	39 (44.3)	**0.008**	14 (15.9)	74 (84.1)	**<0.001**	19 (21.6)	69 (78.4)	**0.001**
Marital status	Unmarried	138 (40.7)	201 (59.3)		117 (34.5)	222 (65.5)		27 (8)	312 (92)	
	Married	36 (57.1)	27 (42.9)	**0.016**	15 (23.8)	48 (76.2)	0.097	19 (30.2)	44 (69.8)	**<0.001**
Religion	Hinduism	158 (43.9)	202 (56.1)		119 (33.1)	241 (66.9)		42 (11.7)	318 (88.3%)	
	Other than Hinduism	16 (38.1)	26 (61.9)	0.473	13 (31)	29 (69)	0.784	4 (9.5%)	38 (90.5%)	0.680
Ethnicity	Brahmin/Chettri	115 (39.8)	174 (66.2)		108 (37.4)	181 (62.6)		29 (10)	260 (90)	
	Other than Brahmin/Chettri	59 (52.2)	54 (47.8)	**0.024**	24 (21.2)	89 (78.8)	**0.002**	17 (15)	96 (85)	0.156
Education level	1st, 2nd, and 3rd year	50 (29.6)	119 (70.4)		63 (37.5)	106 (62.5)		16 (9.5)	153 (90.5)	
	4th year	124 (53.2)	109 (46.8)	**<0.001**	69 (29.6)	164 (70.4)	0.106	30 (12.9)	203 (87.1)	0.289
Family history	Yes	2 (25.0)	6 (75.0)		8 (100)	0 (0)		2 (25)	6 (75)	
	No	172 (43.7)	222 (56.3)	0.2920	132 (33.5)	262 (66.5)	**0.046**	44 (11.2)	350 (88.8)	0.224
Testicular abnormality	Yes	34 (66.7)	17 (33.3)		10 (19.6)	41 (80.4)		11 (21.6)	40 (78.4)	
	No	140 (39.9)	211 (60.1)	**<0.001**	182 (34.8)	229 (65.2)	**0.031**	35 (10)	316 (90)	**0.015**
Sources of information	Health worker	56 (38.4)	90 (61.6)	**0.132**	55 (37.7)	91 (62.3)	0.119	31 (21.2)	115 (78.8)	**<0.001**
	Sex education	52 (37.4)	87 (62.6)	0.084	52 (37.4)	87 (62.6)	0.156	29 (20.9)	110 (79.1)	**<0.001**
	Mass media	116 (41.9)	161 (58.1)	0.397	107 (38.6)	170 (61.4)	**<0.001**	37 (13.4)	240 (86.6)	**0.0073**
	Parents and teachers	28 (20.6)	108 (79.4)	**<0.001**	51 (37.5)	85 (62.5)	0.154	20 (14.7)	116 (85.3)	0.142

%: percentage; *p* value of less than 0.05 is considered significant.

**Table 7:** Logistic regression analysis for sociodemographic factors associated with KAP regarding testicular cancer and testicular self-examination.

	Level of knowledge		Level of attitude		Level of practice	*n* = 402
Variables	AOR (95% CI)	*p* value	AOR (95% CI)	*p* value	AOR (95% CI)	*p* value
Age in group (25 years vs. above 25 yrs^∗^)	1.122 (0.621-2.028)	0.703	0.362 (0.186-0.706)	**0.003**	0.396 (0.191-0.821)	**0.013**
Marital status (unmarried^∗^ vs. married)	4.516 (1.962-10.397)	**<0.001**	0.524 (0.241-1.141)	0.104	0.347 (0.156-0.775)	**0.010**
Religion (Hinduism vs. other^∗^ religions)	1.552 (0.637-3.779)	0.333	0.724 (0.314-1.669)	0.449	0.478 (0.137-1.668)	0.247
Ethnicity (Brahmin/Chettri vs. others^∗^)	2.606 (1.443-4.709)	**0.002**	0.399 (0.218-0.728)	**0.003**	0.593 (0.277-1.272)	0.179
Education (1st, 2nd, 3rd year vs. 4th year^∗^)	2.568 (1.549-4.258)	**<0.001**	0.895 (0.554-1.445)	0.650	0.928 (0.437-1.974)	0.847
Sources of information, health worker (yes vs. no^∗^)	0.389 (0.571-2.671)	0.337	2.656 (0.480-14.697)	0.263	0.373 (0.551-2.522)	0.312
Sex education (yes vs. no^∗^)	1.457 (0.221-9.622)	0.696	0.445 (0.083-2.376)	0.343	0.774 (0.127-4.728)	0.781
Mass media (yes vs. no^∗^)	1.276 (0.732-2.224)	0.389	2.346 (1.328-4.143)	**0.003**	0.955 (0.373-2.447)	0.924
Parents and teachers (yes vs. no^∗^)	0.551 (0.024-0.127)	**<0.001**	1.956 (1.162-3.291)	**0.012**	1.407 (0.623-3.177)	0.380
Family history (yes vs. no^∗^)	2.410 (0.266-21.835)	2.410	—	—	0.314 (0.050-1.975)	0.217
Testicular abnormality (yes vs. no^∗^)	12.827 (4.850-33.924)	**<0.001**	0.426 (0.189-0.960)	**0.039**	0.868 (0.3422.204)	0.766

^∗^Reference group. AOR: adjusted odds ratio; CI: confidence interval. *p* value of less than 0.05 is considered significant.

**Table 8:** Correlation between KAP scores.

Variables	Correlation coefficient (*r*)	*p* value
Knowledge-attitude	-0.301	**<0.001**
Knowledge-practice	0.093	0.061
Practice-attitude	0.100	**0.045**

^∗^Correlation is significant at the 0.05 level (2-tailed).

## Data Availability

The data and materials that are used in this study are available from the corresponding author.

## Abbreviations

TC: Testicular cancer
TSE: Testicular self-examination
KAP: Knowledge, attitude, and practice
SD: Standard deviation.
